The article "Finite Element Prediction on Fracture Load of Femur with Osteogenesis Imperfecta under Various Loading Conditions" was retracted in 2023. Reasons: signs of a paper mill; suspected computer-generated content; unreliable results or conclusions; concerns about the data.

# Finite Element Prediction on Fracture Load of Femur with Osteogenesis Imperfecta under Various Loading Conditions

**DOI:** 10.1155/2022/8722333

**Published:** 2022-01-21

**Authors:** Soh Bua Chai Wanna, Khairul Salleh Basaruddin, Fauziah Mat, Mohd Hanafi Mat Som, Abdul Razak Sulaiman

**Affiliations:** ^1^Faculty of Electronic Engineering Technology, Universiti Malaysia Perlis, 02600 Pauh Putra, Perlis, Malaysia; ^2^Faculty of Mechanical Engineering Technology, Universiti Malaysia Perlis, 02600 Pauh Putra, Perlis, Malaysia; ^3^Sport Engineering Research Center, Universiti Malaysia Perlis, 02600 Pauh Putra, Perlis, Malaysia; ^4^Department of Orthopaedics, School of Medical Science, Universiti Sains Malaysia, 16150 Kubang Kerian, Kelantan, Malaysia

## Abstract

Osteogenesis Imperfecta (OI) is an inherited disorder characterized by extreme bone fragility due to collagen defects. It is an incurable disease. Bone fractures can occur frequently without prior notice, especially among children. Early quantitative prediction of fracture loads due to OI tends to alert patients to avoid unnecessary situations or dangerous conditions. This study is aimed at investigating the fracture loads of femur with OI under various types of loading. Ten finite element models of an OI-affected bone were reconstructed from the normal femur with different bowing angles ranging from 7.5 to 30.0°. The boundary conditions were assigned on an OI-affected femoral head under three types of load: medial-lateral impacts, compression-tension, and internal-external torsions, and various loading direction cases that reflect the stance condition. The fracture load was examined based on the load that can cause bone fracture for each case. The results show that the loads bearable by the femur before fracture were decreased with respect to the increase of OI bowing angles in most of the loading cases. The risk of fracture for the femur with OI was directly proportional to the increase of bowing angles in the frontal plane. This study provides new insights on fracture load prediction in OI-affected bone with respect to various loading types, which could help medical personnel for surgical intervention judgement.

## 1. Introduction

Osteogenesis Imperfecta (OI) is a rare bone disease affecting the bone in a manner that increases the likelihood of fractures. Byers and Steiner suggested that this disease appears to affect between 1 in 5,000 and 1 in 10,000 of the population [1]. Among infants, the prevalence of OI is between 1 in 15,000 and 1 in 20,000 [2]. However, many are not aware of the occurrence of the disease unless it befalls their family members. A gene mutation that causes permanent changes in collagen structure is the main cause of OI [3]. This disease can be classified into four main types (type I–IV) according to a classification system study by Silence et al. [4]. Type I is the mildest form of OI with apparent blue sclera and little bone deformity. Type II is the most severe type, where death normally occurs either in the uterus or within 24 hours of birth. People with type III OI experience frequent fractures and display features such as triangular face, scoliosis, brittle teeth, and possible hearing loss. Type IV is the moderate type of OI with common features such as short stature and mild to moderate scoliosis. Damaged or degraded collagen in the bone as a direct effect of the gene mutation results in low bone mass and high bone fragility [5, 6]. These conditions lead to repeated fractures in OI patients.

The article "Finite Element Prediction on Fracture Load of Femur with Osteogenesis Imperfecta under Various Loading Conditions" was retracted in 2023. Reasons: signs of a paper mill; suspected computer-generated content; unreliable results or conclusions; concerns about the data.

Repeated fractures will create difficulty in attempting daily basic movements, especially for children. Thus, early prediction of fracture risk using a clinical and computer-based approach with finite element analysis (FEA) could assist in this issue [7, 8]. Early detection of fracture risk would allow for better medical care, reduce pain, prevent any unforeseen circumstances that could lead to other health issues, and help patients participate in activities of daily living (ADL). Mechanical OI bone modeling studies are basically aimed at helping predict fractures in OI-affected bone through a continuum mechanics-based model via FEA. The use of FEA in biological structures was reported as one of the better-established platforms for conveying complex and convoluted biological structures through a simulation-based approach. This allows for advanced improvement in medical research by predicting and helping calculate the possibility of fracture. Previous researches by Caouette et al. [8], Frit et al. [9], and Fan et al. [10] were aimed at predicting fracture risk in long bones of OI patients. Caouette et al. [8] used FEA to model OI-affected bone in their study in order to predict fracture risk in OI patients with tibia deformity, where seven different boundary conditions were applied for various types of loading cases, identified as two-leg hopping; external and internal forces of tibia torsion; and medial, lateral, posterior, and anterior sections. The findings proved that there is a correlation between fracture risk and tibial bowing, but the conclusion is only applicable in vertical compressive loading. Fritz et al. [9] explained the relationship between fracture risk and OI bowing angles using a standard femur which was later modified to match the morphology of a patient diagnosed with type I OI. The fracture risk was specifically examined in seven gait cycle phases of loading response: mid stance, terminal stance, preswing, initial swing, mid swing, and terminal swing. Results from the study suggest that there is no risk of fracture during normal gait. On the other hand, Fan et al. [10] conducted FEA of the femur to investigate the influence of deformity in the stress/strain relationship with respect to the 10% gait cycle. The results indicate that the stress/strain distribution increases as the severity of bowing angles increased. In severe cases, where the stress/strain drastically increases and is expected to be greater than the stress threshold, it was postulated that fracture might occur in that particular area. The authors' previous studies also investigated the similar cases, focusing the OI bone fracture due to load of ADL [11] and different load directions [12]. Overall, these studies were aimed at unveiling the risk of fracture with the sole purpose of providing preventive care for OI patients.

The article "Finite Element Prediction on Fracture Load of Femur with Osteogenesis Imperfecta under Various Loading Conditions" was retracted in 2023. Reasons: signs of a paper mill; suspected computer-generated content; unreliable results or conclusions; concerns about the data.

However, what remains unclear is how the load direction in the femoral head of OI-affected bone could contribute to the fracture risk. The hip joint connects to the axial skeleton with long bones and is the primary connection that assists in normal mobility during everyday life. The effect of load direction can greatly influence the severity of hip fractures, especially in the femoral head. Several research studies on the influence of force direction on the femoral head were conducted; however, none focused on the OI-affected bone [13–15]. Thus, in the present study, we predicted the fracture load of OI bone, which is the optimum load bearable by the femur with OI before fracture using finite element analysis under various loads consisting of compression, tensile, torsional, and impact loads, as well as loads applied in a standing configuration in the sagittal and frontal planes.

## 2. Materials and Methods

### 2.1. Geometrical Model of OI-Affected Bone

The “standardized femur” (SF) model was first obtained from the BioMed Town website proposed by Viceconti et al. to make it available for download [16]. The length of the SF is 409.4 mm. The SF was then imported into Ansys ver. R18.1, a software package for conducting FEA. The design modeler was used to divide the SF into two parts: the femoral head and the femoral shaft. The original SF was imported in one full part; thus, its separation into two parts for the simulation was considered. At the origin, a perpendicular line with 45° was drawn in the *Z*-plane to divide the femoral head and femoral shaft. Once divided, the femoral head and femoral shaft are bonded with same mechanical properties. After separating the femoral head and femoral shaft, the SF was then reconstructed in the OI model with ten different bowing angles.

The article "Finite Element Prediction on Fracture Load of Femur with Osteogenesis Imperfecta under Various Loading Conditions" was retracted in 2023. Reasons: signs of a paper mill; suspected computer-generated content; unreliable results or conclusions; concerns about the data.

A radiography image of a CT scan obtained from Hospital Universiti Sains Malaysia from an enrolled OI patient provided guidance for reconstructing the finite element OI model. The tangent rule was used to deform SF to ten different bowing angles ranging from 7.5 to 30.0° in 2.5° increments. The length of the bone was measured and divided in half, and the value was used as a reference point for the deformed bone to represent the OI-affected bone geometry. Nodal displacement was used to describe deformation. A node was selected to mark the center of the SF model, and the node was displaced. This was repeated for the next nine SF models with different bowing angles. The displacement value varies according to the aforementioned equation, which is used to diversify the bowing angles. The SF models were altered by matching them with CT images of OI-affected bone in the frontal plane. The radiograph image was used as a template to fit the SF. Ten bowing angles were then reconstructed, where a 17.5° bowing angle provided the best fit with the CT image, whereas the remaining nine bowing angles were used to model variations in the OI bone bowing angles. These models serve as guidelines for determining fracture loads for various bowing angles. The constraint was set at the femoral head, medial condyles, lateral condyles, and intercondylar fossa of the femur.  Figure 1(a) shows a radiograph image of an enrolled OI patient, and Figure 1(b) shows the reconstructed OI finite element model.  Figure 2 shows examples of bowing angle at 10.0°, 15.0°, 20.0°, 25.0°, and 30.0°.

### 2.2. Meshing and Material Properties

The SF was meshed using 22,064 nodes and 12,224 elements with a tetrahedron patch conforming method when the element size was set to 3 mm. Mechanical properties were assigned based on the work conducted by Fan et al. [17, 18] by performing nanoindentation tests on femur bone samples. Thus, the same mechanical properties were applied in this simulation; the SF was defined as isotropic and linear elastic with Young's modulus of 19 GPa and Poisson's ratio of 0.3.

### 2.3. Boundary Conditions

The boundary conditions were assigned to the OI-affected femur in order to investigate the effect of the loading direction on bone fracture for various load impacts. Lateral and medial impacts, compression and tension, and external and internal torsion loads were applied on the surface of the femoral head along the direction shown in Figure 3. For the load direction, a total of 14 loading conditions were considered, as listed in Table 1 [13, 14]. In the stance condition, the first eight conditions correspond to a force direction that was tilted from 3 to 24° in the frontal plane and from 0 to 18° in the sagittal plane. In the frontal plane, the angle moves from anterior to posterior, while in the sagittal plane, the direction points from the lateral to medial. Another six conditions involve a combination of these two planes. For all loading conditions, the constraint was set at the medial condyles, lateral condyles, and intercondylar fossa of the femur, and the force was applied on the femoral head.

The article "Finite Element Prediction on Fracture Load of Femur with Osteogenesis Imperfecta under Various Loading Conditions" was retracted in 2023. Reasons: signs of a paper mill; suspected computer-generated content; unreliable results or conclusions; concerns about the data.

### 2.4. Fracture Load Assessment

Fracture load was assessed to fulfill the main objective, which is to identify the optimum load bearable by the femoral head with OI before fracture under various load types. A fracture strength of 115 MPa was obtained from the nanoindentation test, which reflects the 75% strength of normal adolescent femurs and the strength of the OI bone [9].

## 3. Results

### 3.1. Fracture Load in OI-Affected Bone under Different Load Types

Figure 4(a) shows the fracture load for bowing angles for medial and lateral impacts in the sagittal plane. Overall, the fracture load increased for both conditions of all bowing angles. However, the increment in the medial case was higher, with an average difference of 838.26 N compared to the lateral case. The highest fracture load in the medial impact was 1232.7 N and the lowest was 864.2 N. Lateral impact exhibited the greatest fracture load of 1073.4 N and the lowest fracture load of 846.80 N. The fracture load does not show a large difference between the two cases for the first two bowing angles and starts to show a wider gap when it reached a bowing angle of 12.5°. The fracture load in both cases increases as the bowing angles increase, and greater differences are seen between two cases.

Moreover, Figure 4(b) shows the fracture load for ten bowing angles under compression and tension loads. These two cases behave oppositely in marked contrast to the medial and lateral load cases. The fracture load decreased as the bowing angle increased from 7.5 to 22.5° and started to marginally increase for the last three bowing angles in the compression load case. Tensile loads produced the same behavior, except for the increase in fracture load starting at a bowing angle of 25.0°. The maximum loads required for fracture were 3674 N and 2876.75 N and the minimum were 3192 N and 2078.64 N for compression and tensile loads, respectively.

Figure 4(c) shows the fracture load for external and internal torsions acting on the femoral head in the sagittal plane. In external load cases, the fracture load increased as the bowing angles increased. In contrast to external torsion, the internal torsion produces opposite behavior. The fracture load decreases as the bowing angle increases. The highest fracture load was 240.5 N·mm in external rotation and 248.2 N·mm for internal rotation.

The article "Finite Element Prediction on Fracture Load of Femur with Osteogenesis Imperfecta under Various Loading Conditions" was retracted in 2023. Reasons: signs of a paper mill; suspected computer-generated content; unreliable results or conclusions; concerns about the data.

### 3.2. Fracture Load of OI-Affected Bone under Various Loading Conditions

On the other hand, Figure 5(a) shows the fracture load as a function of the bowing angles in the sagittal plane. The fracture load when the load direction was 3° and 8° decreased minimally. In contrast, when the load direction was 24°, the fracture load increased as the bowing angle increased; the greatest fracture loads were 4350 N, 6105 N, and 5200 N. When the load direction was 3° and 8°, there were large differences in the fracture loads for the first four bowing angles. However, those gaps became smaller as the bowing angles increased.

Figure 5(b) shows the fracture load at all bowing angles in a frontal plane. The trend was the same for the 3° posterior and 10° anterior load directions, as indicated by the OI-affected bone models in the frontal plane. The fracture load decreased for the first three bowing angles, remained fairly constant for the next three bowing levels, and increased for the last four bowing angles. On the other hand, given the load at 18° anterior, there was a steady increment in the fracture load for all bowing angles. The highest fracture loads recorded at 3°, 10°, and 18° directions were 2853 N, 3148 N, and 3556 N, respectively.

Figure 5(c) shows the load direction in the sagittal and frontal planes as a function of the bowing angle. Overall, the trends are similar for all six conditions. There was a minimal decrease in the fracture load for the first six bowing angles, and the fracture load remained nearly constant before increasing. The largest load ranged from 2136 to 3211 N, while the smallest load ranged from 1806 to 2160 N. The incline was found to be rather high when the load direction was at larger medial angles (12° and 18°) compared to smaller medial angles (6° and 8°).

## 4. Discussion

Various external loads, such as impact, torsional, compression, and tension, can cause injury and fracture to the OI patient's bone. In the sagittal plane, the fracture load for medial and lateral loads increases as the bowing angles increase in the OI models. The load required for all models to encounter fracture in the medial direction is higher compared to the load in the lateral direction. This could be related to the anatomical location of the femur bone. In the sagittal plane, the medial impact originates from the inner part of the body. In contrast, lateral impact originates from an outer part of the body. Therefore, a bone is more vulnerable to fracture due to a lateral impact. The external forces will affect bone strength. In relation to our study, Caouette et al. [8] also reported similar findings. The fracture load for the medial impact is higher than that for the lateral impact in the sagittal plane. The internal torsional fracture torque increases with increasing bowing angle. On the contrary, the external torsion fracture torque decreases as the bowing angles increase. Torsional loading will produce a stress distribution over the cross-sectional area, as shown by Grutter et al. in their cadaveric study [19], which is consistent with the results in this study. The femoral neck is the weakest part of the femur due to its small cross-sectional area and is the most frequently injured part of the femur [20]. Hence, when a torsional load was applied on the femoral head, the femoral neck was unable to support the twisting effect. Compared to other load conditions, an axial load will produce a uniform stress throughout the cross-section of the object.

The article "Finite Element Prediction on Fracture Load of Femur with Osteogenesis Imperfecta under Various Loading Conditions" was retracted in 2023. Reasons: signs of a paper mill; suspected computer-generated content; unreliable results or conclusions; concerns about the data.

On the contrary, the relationship between the fracture loads for compression and tension loads is different for various bowing angles. The stress decreases as both conditions approach larger deformed models. The compressive force is the main source of fracture in bones [15]. Bones become stronger when given a compressive force, and they are more delicate due to an applied tensile force [21]. This statement is consistent with the findings from this study. It appears that the required compression loading for the model to reach fracture is greater than the required tension loading. The greatest load models were capable of bearing compressive and tensile loads of 3674 N and 2876.75 N, respectively.

The optimum fracture load for various load directions suggests that the maximum load required for fracture is 4350 N, 6105 N, and 5200 N in the sagittal plane of the femoral head when the load direction was 3°, 8°, and 24°, respectively. Changes in these trends were obvious given the differential load angles in the sagittal plane; the trend changed with load angle. Given the medial load direction of 3° and 8°, the fracture load decreased when the bowing angle in the OI model increased. As the load direction moves toward the medial direction of the body at 24°, the fracture load started to show random changes in which the fracture load increased as the bowing angle increased. Nonetheless, we attempted to clarify this situation by exploring other possible angles that may possibly exhibit similar trends, even though these possible angles were not mentioned in the reference journal. Angles of 3°, 8°, and 24° were used in this study based on previous research [13, 14]. Hence, to explain the situation, we also explored angles of 16° and 20°, and the results can be used to explain why the trend suddenly changes from an inversely proportional dependence to a linear dependence. The latter trend indicates that as the angles move toward the medial segment of the body, the fracture load began changing from the least deformed bowing angle to the most deformed bowing angle. This would clearly explain the transformation of the trend. During simulation, all models experienced the greatest fracture at the bowing part of the femoral shaft at different loads where all the red contours accumulated. This shows that as the femoral head is given a certain load, the middle part of the femur will be unable to bear the load given all the conditions and will fracture first. In the frontal plane, the trend was similar for all three conditions. The fracture load is decreased as the bowing angle increases until it reached its maximum load when the bowing angle was 20°. The fracture load started to increase slightly for greater bowing angles. Joyce et al. investigated the force direction due to impact from a fall and atraumatic loading; their results suggest that the risk of hip fracture is greatly affected by the force direction, which is determined by fracture load [5]. The results show that the greatest average fracture load was 1797 N when the angle with respect to the femoral head was 70° from the shaft and 55° between the femoral head toward the anterior direction in the fall configuration.

The article "Finite Element Prediction on Fracture Load of Femur with Osteogenesis Imperfecta under Various Loading Conditions" was retracted in 2023. Reasons: signs of a paper mill; suspected computer-generated content; unreliable results or conclusions; concerns about the data.

On the other hand, for atraumatic loading, the lowest fracture load was 2792 N whereas the greatest fracture load was 5148 N when the angles were set in between the femoral head in the sagittal and coronal planes [5]. In comparison to our finding, the highest fracture load was 6105 N when the angle was set at 24° in the sagittal plane, 3556 N at 10° in the frontal plane, and 3211 N when the planes were combined. In comparison to our finding which focuses on the stance of OI patients, the fracture load required was rather explainable since, as no movement was required during this phase, the difference was between the fall and atraumatic conditions, and their study focused on normal subjects. Force impact on the femoral head causes either compression or tension in the body, leading to injury. In the frontal plane, as the force direction moves to the posterior of the body, the risk of fracture is lower compared to the case where the body started to move anteriorly. The hip joint begins to move anteriorly just before reaching toe off, indicating that an OI patient should take better precautions because the possibility of fracture is greatest. As the angle increases from 3 to 24° in the same sagittal plane, the trend changes for different bowing angles. In the case of smaller variations in bowing angles, the smallest bone deformity of 7.5° required the greatest fracture load, which would explain the lower fracture risk in the stance phase. However, when the force was applied at a larger angle and was targeted at the femoral head, the 7.5° angle in the SF model required the lower fracture load. In contrast, when the direction of force was applied at a smaller angle, the fracture load minimized at the maximum bowing angle (30°), while the fracture load was larger when the load was applied at a larger angle.

The article "Finite Element Prediction on Fracture Load of Femur with Osteogenesis Imperfecta under Various Loading Conditions" was retracted in 2023. Reasons: signs of a paper mill; suspected computer-generated content; unreliable results or conclusions; concerns about the data.

## 5. Conclusion

The main purpose of the current study was to determine the fracture loads of the femur with OI for variations in the bowing angle ranging from 7.5 to 30.0° under different loading conditions. The results of the FEA show that the fracture loads were gradually increased with respect to the increase of bowing angles for medial-lateral impact and external torsion directions, whereas the compression and tension loads made no significant difference to the fracture loads. One of the most significant findings to emerge from this study is that the fracture load was found decreased as the bowing angle increases for internal torsion and standing load configuration in frontal and sagittal planes. These findings enhance our understanding on the optimum load bearable by the femur with OI before fracture is reduced due to increases of bowing angle under certain load conditions. Therefore, early prediction of fracture risk in OI patients is important as it raises awareness for family members and orthopedics to prepare for both unpredictable consequences and the best available treatment methods. Variations in the angles on the femoral head in the sagittal and frontal planes and their effects on the possibility of fracture provide medical personnel with better information for assisting OI patients to improve their mobility and prevent fracture. Overall, this study provides vital information on the force direction acting on the femoral head and helps predict fracture risk in particular configurations.

## Figures and Tables

**Figure 1:** Reconstruction of geometrical model of OI bone: (a) CT image of OI patient; (b) reconstructed finite element model of OI-affected bone.

**Figure 2:** Examples of OI-affected bone models with (a) 10°, (b) 15°, (c) 20°, (d) 25°, and (e) 30° bowing angles.

**Figure 3:** Loadings on femoral head: (a) lateral and medial impacts; (b) compression and tension; (c) external and internal torsions.

**Figure 4:** Fracture load as a function of the bowing angle for different load types: (a) fracture load in medial and lateral impacts; (b) fracture load in compression and tensile stresses; (c) fracture load in external and internal torsions.

The article "Finite Element Prediction on Fracture Load of Femur with Osteogenesis Imperfecta under Various Loading Conditions" was retracted in 2023. Reasons: signs of a paper mill; suspected computer-generated content; unreliable results or conclusions; concerns about the data.

**Figure 5:** (a) Fracture load in the frontal plane; (b) fracture load in the sagittal plane; (c) fracture load in the frontal and sagittal planes.

**Table 1:** Variation of load direction in the frontal and sagittal planes.

Load cases	Frontal plane	Sagittal plane	Frontal + sagittal
1	3° medial	—	—
2	8° medial	—	—
3	16° medial		
4	20° medial		
5	24° medial	—	—
6	—	Neutral	—
7	—	3° posterior	—
8	—	18° anterior	
9	—		8° medial–4.5° anterior
10		—	8° medial–8° anterior
11	—	—	12° medial–9° anterior
12	—	—	12° medial–13.5° anterior
13	—	—	18° medial–4.5° anterior
14	—	—	18° medial–13.5° anterior

## Data Availability

The data used to support the findings of this study are available from the corresponding author upon request.
